# Strongyloidiasis in Africa: Systematic Review and Meta-Analysis on Prevalence, Diagnostic Methods, and Study Settings

**DOI:** 10.1155/2020/2868564

**Published:** 2020-11-15

**Authors:** Tadesse Hailu, Endalkachew Nibret, Arancha Amor, Abaineh Munshea

**Affiliations:** ^1^College of Medicine and Health Sciences, Bahir Dar University, Bahir Dar City, Ethiopia P.O. Box 79; ^2^Biology Department, Science College, Bahir Dar University, Bahir Dar City, Ethiopia P.O. Box 79; ^3^Mundo Sano Foundations, Madrid, Spain

## Abstract

**Background:**

*Strongyloidiasis* is an intestinal parasitic infection mainly caused by *Strongyloides stercoralis*. Although it is a predominant parasite in tropics and subtropics where sanitation and hygiene are poorly practiced, the true prevalence of s*trongyloidiasis* is not known due to low-sensitivity diagnostic methods.

**Objective:**

This systematic review and meta-analysis is aimed at determining the pooled prevalence of s*trongyloidiasis* in African countries, stratified by diagnostic methods, study settings, and patients.

**Methods:**

Cross-sectional studies on strongyloidiasis published in African countries from the year 2008 up to 2018 in PubMed and Google Scholar databases and which reported at least one *Strongyloides* spp. infection were included. Identification and screening of eligible articles were also done. Articles whose focus was on *strongyloidiasis* in animals, soil, and foreigners infected by *Strongyloides* spp. in Africa were excluded. The random effects model was used to calculate the pooled prevalence of s*trongyloidiasis* across African countries as well as by diagnostic methods and study settings. The heterogeneity between studies was also computed.

**Result:**

A total of 82 studies were included. The overall pooled prevalence of s*trongyloidiasis* was 2.7%. By individual techniques, the pooled prevalence of strongyloidiasis was 0.4%, 1.0%, 3.4%, 9.3%, 9.6%, and 19.4% by the respective direct saline microscopy, Kato-Katz, formol ether concentration, polymerase chain reaction, Baermann concentration, and culture diagnostic techniques. The prevalence rates of strongyloidiasis among rural community, school, and health institution studies were 6.8%, 6.4%, and 0.9%, respectively. The variation on the effect size comparing African countries, diagnostic methods, study settings, and patients was significant (*P* ≤ 0.001).

**Conclusions:**

This review shows that strongyloidiasis is overlooked and its prevalence is estimated to be low in Africa due to the use of diagnostic methods with low sensitivity. Therefore, there is a need for using a combination of appropriate diagnostic methods to approach the actual *strongyloidiasis* rates in Africa.

## 1. Introduction

*Strongyloides stercoralis* is one of the soil-transmitted helminths (STHs) that cause strongyloidiasis. There are more than 60 species in the genus which parasitize the duodenum of the small intestine of humans and domestic mammals [1]. Only two species *S. stercoralis* and *S. fuelleborni* are known to infect human beings. *Strongyloides stercoralis* is distributed in tropical and subtropical areas whereas *S. fuelleborni* infection is found in Papua New Guinea and sporadically in Africa [2].

The true prevalence of strongyloidiasis is underestimated and underreported due to the use of diagnostic methods with poor sensitivity [3]. An estimated 370 million strongyloidiasis occur globally [4], being 90% of them in sub-Saharan Africa, Southeast Asia, Latin America, Oceanian countries, and the Caribbean islands and is related to poor sanitation and hygiene practices [5]. Studies showed that high numbers of strongyloidiasis occur among children [6] and immunocompromised individuals [7]. Several factors including malnutrition, autoimmune diseases, and taking corticosteroid drugs that impaired the immune system may contribute for the high prevalence of *strongyloidiasis* [8].

In developing countries, the risk of acquiring strongyloidiasis is higher in rural dwellers, having low socioeconomic status [9] and poor sanitation infrastructures [10]. Infection ranges from asymptomatic to life-threatening clinical manifestations depending on the level of immunity [11]. The infection appears when the filariform larva enters the human body through skin penetration and crosses the lung during larva migration, and the adult reaches the small intestine. The larvae may cause skin rashes, dry cough, and recurrent sore throat whereas the adult stage of the parasite may also cause abdominal pain, loss of appetite, diarrhea, blood in stool, epigastric pain, and bloating, but most frequently, the infection is asymptomatic [12].

Strongyloidiasis is detected by microscopic-based diagnostic methods like direct saline microscopy (DSM) [3], formol ether concentration technique (FECT) [13], Baermann concentration technique (BCT) [14], agar plate technique (APT) [15], and immunological [16] and molecular-based techniques [17].

The Baermann concentration technique may increase the detection rate of strongyloidiasis by 3.6-4 times compared to the FECT or DSM technique [18]. In the same way, serological assays [16] and real-time polymerase chain reaction (RT-PCR) techniques have shown to be more sensitive diagnostic tools for *S. stercoralis* detection [17].

The sensitivity of BCT, APT, RT-PCR, and ELISA is good, but not enough. Moreover, they have limitations for application in countries of poor resource in Africa. Because of that, a combination of techniques is the recommended approach for diagnosing the infection. Therefore, this systematic review and meta-analysis is aimed at providing an overview of the prevalence of strongyloidiasis across African countries, stratified by diagnostic methods, study settings, and patients.

## 2. Materials and Methods

A search on the databases PubMed and Google Scholar was done for studies written in English from the year 2008 up to 2018. Keywords used in the search were “Strongyloidiasis,” “*Strongyloides*,” “*Strongyloides stercoralis*,” and “Soil-transmitted helminths” in each African country. The search for electronic data of studies was conducted between July 2019 and August 2019. Identification, screening, and checking the eligibility and the inclusion of the relevant studies were done following the preferred reporting items for systematic reviews and meta-analyses (PRISMA) (Figure 1). The articles extracted from the two databases were first screened to remove duplication. Furthermore, the articles were screened by reading their abstracts and the full articles and then the articles which did not investigate the prevalence of strongyloidiasis.

### 2.1. Inclusion Criteria

All cross-sectional studies from 2008 to 2018 conducted in African countries among patients or any participants in Africa and diagnosed by DSM, KK, FECT, BCT, culture, PCR, or a combination of these diagnostic techniques and obtained at least one positive for *Strongyloides* spp. were included. Including only PubMed and Google Scholar databases was the limitation.

### 2.2. Exclusion Criteria

All studies on strongyloidiasis in animals, soil, foreigners in African countries or imported cases, nondefined study population, sample sources other than stool, analysis of *S. stercoralis-*positive cases only, method comparisons, case studies, cohort studies, duplications, articles conducted before the year 2008, and review articles done in African countries were excluded. The suitability of all studies according to the defined criteria was judged independently by two different authors. Any differences in judgment were resolved by discussion among the authors.

For each selected paper, the following information was recorded: number of infected individuals, number of examined individuals, country name, types of diagnostic method used, study setting where date were collected, and types of disease recorded in health institution. The pooled prevalence of strongyloidiasis in African countries as well as by each diagnostic method, study settings, and among patients was computed using a random effects model.

The meta-analysis was performed using comprehensive meta-analysis 2.2 software (Biostat Inc., Englewood, NJ, USA). The pooled overall prevalence of strongyloidiasis at 95% confidence interval (CI) in African countries was calculated using a random effects model. The pooled prevalence of strongyloidiasis by diagnostic methods, study settings, and patients was calculated in the subgroup analysis. The forest plot was reported, and separate meta-analyses were performed to evaluate the effect of diagnostic methods, study settings, and patients in health institutions with strongyloidiasis. Heterogeneity (the difference between studies) by country, diagnostic methods, study settings, and among patients was assessed using Cochran (*Q*) value, *P* value, and *I*^2^ and visual inspection of the forest plot. The level of significance for all tests was *P* ≤ 0.001. Publication bias that occurs in published studies was checked by considering effect size symmetry on funnel plot (a scatter plot of estimates). Absence of bias is presented by shape like a funnel.

## 3. Result

A total of 208 (90 from PubMed and 118 from Google Scholar databases) studies were identified. One hundred sixty-three studies were screened and recorded after duplications removed. One hundred twenty-one studies were found to be eligible after full-text assessment, and finally, 82 studies were included in qualitative analysis (Figure 1).

### 3.1. Prevalence of Strongyloidiasis

Twenty African countries having strongyloidiasis research reports and fulfilling the inclusion criteria were involved with the total participants being 96,069 (Table 1).

Among the 82 studies in Africa, the prevalence of strongyloidiasis ranged from 0.1% in a study conducted in Sudan [87] to 27.1% in Côte d'Ivoire [26] (Table 1). All studies in Côte d'Ivoire used a combination of two or three diagnostic techniques including PCR, BCT, and culture techniques. One of the two studies from Mozambique also used combination of FECT, BCT, and PCR reporting a prevalence rate of 48.51% [59]. The prevalence rate 17.4% in Rwanda was reported using agar plate culture among community dwellers [84]. The fourth highest prevalence 10.21% (92-96%) of strongyloidiasis was from Tanzania. All the five studies [89–93] conducted in Tanzania used BCT as diagnostic method, and three of which studies used PCR [90], FECT [93], or culture [94] (Table 1).

In Ethiopia, a relatively high number of participants 44,638 (45.1%) were included (Table 1) and the total pooled prevalence of strongyloidiasis was 1.1% (1.0-1.2) (Figure 2). Most of the studies (13/18; 72.2%) used FECT, whereas four studies (22.2%) used DSM as a means of diagnosis. The majority of the studies (12/18: 66.7%) were conducted among patients visiting the health institutions for different ailments (Table 1).

In Nigeria, a total of 14,294 (14.8%) study participants were involved in 23 (27.7%) studies (Table 1). The pooled prevalence of strongyloidiasis in Nigeria was 4.9% (4.5-5.2%) (Figure 2). Nineteen (82.6%) and three (13.0%) of the studies used FECT and DSM diagnosis in Nigeria, respectively. Only one study used culture diagnostic method. In addition, 15 (65.2%) and eight (34.8%) studies were conducted among school-age children and patients, respectively (Table 1).

Low pooled prevalence of strongyloidiasis was reported from studies conducted in Sudan (0.14%) [87], Zambia (0.5%) [97], and Burkina Faso (0.5%) [22]. Among studies conducted in Sudan, one study conducted using DSM [88] and the other by FECT [87] had low sensitivity to strongyloidiasis detection. The studies conducted in Burkina Faso and Zambia used DSM as a diagnostic method (Table 1).

The forest plots (Figure 2) indicated the pooled prevalence of strongyloidiasis among 82 studies in Africa which was 3.4% (95% CI: 2.0-5.5%) using random effects model. The highest pooled prevalence 22.6% of strongyloidiasis was recorded in Côte d'Ivoire followed by Mozambique 22.6% (19.6-25.9%), Rwanda 17.4% (14.5-20.9%), and Egypt 15.7% (10.1-23.4%) (Figure 2). The heterogeneity of studies across African countries was high (*Q* = 2782.625, *I*^2^ = 99.317%, *P* ≤ 0.001) (Figure 2).

### 3.2. Diagnostic Methods of Strongyloidiasis

Regarding the diagnostic methods of *S. stercoralis*, most studies (69, 84.15%) used DM, KK, or FECT. Most of the studies (43, 52.4%) used FECT for diagnosing the infection in Africa (Figure 3). Among studies using single diagnostic methods, high pooled prevalence of strongyloidiasis was recorded 19.4% in stool culture followed by 9.6% in PCR and 9.3% in BCT detection methods (Figure 3). The highest pooled prevalence rate 32.8% of strongyloidiasis was obtained by using a combination of BCT, FECT, and PCR diagnostic methods (Figure 3). The low prevalence rates of strongyloidiasis 3.4%, 0.4%, and 1.0% were also obtained using FECT, KK, and DSM diagnostic methods, respectively (Figure 3).

Forest plot (Figure 3) indicated that the pooled prevalence of strongyloidiasis in Africa across different diagnostic methods was 8.0% (95% CI: 3.9-15.9%) using random effects model. Heterogeneity of studies through different diagnostic approaches was high (*Q* = 3497.655, *I*^2^ = 99.696%, *P* ≤ 0.001) (Figure 3).

### 3.3. Strongyloidiasis by Study Settings

Among the total studies, 35 (42.68%) studies were conducted in health institutions followed by 27 (32.93%) in schools and 18 (21.95%) in rural communities (Figure 4).

The forest plot (Figure 4) shows the pooled prevalence of strongyloidiasis across different study settings in Africa using random effects model which was 1.4% (95% CI: 0.5-3.9%). Heterogeneity of studies among the study sites in the African countries was high (*Q* = 1856.455, *I*^2^ = 9.785%, *P* ≤ 0.001) (Figure 4).

### 3.4. *Strongyloidiasis* In Health Institutions

Pooled prevalence rates of 12.2%, 9.7%, and 3.6% of strongyloidiasis were obtained with the respective tuberculosis (TB), human African trypanosomiasis (HAT), and human immunodeficiency virus (HIV) cases (Figure 5).

Forest plot (Figure 5) indicates 2.3% (95% CI: 0.6-7.7%) pooled prevalence of strongyloidiasis among patients across health institutions in Africa using random effects model. Heterogeneity of studies between patients in the African countries was high (*Q* = 83.334, *I*^2^ = 99.440%, *P* ≤ 0.001) (Figure 5).

The funnel plot shows that studies were distributed symmetrically about the combined effect size that showed the absence of publication bias in this review (Figure 6).

## 4. Discussion

The prevalence of strongyloidiasis in Africa is difficult to estimate due to inadequacy of studies and absence of very high-sensitive diagnostic methods. In this review, authors clearly demonstrated that a study conducted with DSM, FECT, and KK methods provided low strongyloidiasis prevalence report in the African continent. This finding is supported by the most widely used diagnostic methods to helminthic infections including DSM, FECT, and KK which most likely fail to detect strongyloidiasis [18]. The justification for the low prevalence rates of strongyloidiasis in African in the current review might be due to the use of traditional methods (FECT, KK, and DSM), very small amount of stool sample used, and one-time stool sample collection which may give false-negative results. Moreover, single stool examination might also compromise the true prevalence of strongyloidiasis detection. For instance, single stool examination using DSM can detect the strongyloidiasis larvae in only 30% of the cases [99]. Furthermore, the intermittent excretion nature of *S. stercoralis* and chronic low-intensity infections which lead to low larval load within the stool may also affect the true prevalence [7]. Generally, most African countries use low-sensitivity diagnostic methods for strongyloidiasis detection since there is a lack of awareness and more sensitive diagnostic methods are costly and difficult to adopt in most African health institutions. As a result, they stick to using FECT and DSM with their limitations [18].

In this review, stool culture, BCT, and PCR are more sensitive methods for the diagnosis of strongyloidiasis. This finding is supported by other previous studies [15, 100]. A combination of two or three of the culture, BCT, and PCR provided better detection rate of strongyloidiasis in stool in the current review. This result agrees with a previous report [6], and better detection of strongyloidiasis was obtained using combination of BCT and other methods [101]. Nevertheless, it should be borne in mind that the sensitivity of such tests is not perfect, especially when it is performed on a single fecal specimen, diarrheic stool, and a very small amount of stool sample. All these might lead to underdiagnosis and underestimation of the true prevalence of strongyloidiasis. Therefore, there is a need to define a standard protocol in terms of diagnostic methods, the amount and consistency of stool specimens, and the frequency of examination of stool specimens for better assessment of strongyloidiasis. Such priority recommendations and elaboration of mapping guidelines should be done by the World Health Organization for strongyloidiasis like the other soil-transmitted helminthic infections and included in the neglected tropical disease (NTD) group.

The prevalence of strongyloidiasis among community dwellers of Africa in the current review was relatively high (6.69%). This is consistent with an earlier report [7]. This high prevalence of strongyloidiasis in a rural community might be due to low sanitation and hygiene practice, limited knowledge on the transmission of *Strongyloides* infection, and absence of adequate water for sanitation and hygiene in the rural communities of African countries [102, 103].

The prevalence of strongyloidiasis among school children was 6.4% (6.0-6.8%) in this review. A considerable similar report among school-age children is also found in a systematic review conducted in Ethiopia [104]. This might be justified firstly by the fact that African children are living in unhygienic environment with poor sanitation practices where most children play with contaminated soil and walk barefoot that increases the probability of the entrance of the filariform larvae in the body [105]. Secondly, most African children are malnourished [106] and this is evidenced by a high prevalence of strongyloidiasis among malnourished children [107]. Thirdly, a high infection rate of strongyloidiasis was seen in immunocompromised children [108].

In this review, the distribution of strongyloidiasis among patients was 2.3% (0.6-7.7%). This result is consistent with 5.1% prevalence among HIV patients in the previous report [7] but lower than 23% among Bolivian patients [108]. The difference might be due to diagnostic method difference and serological test used in addition to coproparasitological test in a study conducted in Bolivia.

In the current review, heterogeneity of studies was high and there was no publication bias. The current heterogeneity finding is consistent, but the publication bias report disagrees with a previous report [109]. The absence of publication bias might be justified as combined effect size in the current studies is distributed symmetrically using funnel plot.

Unlike other soil-transmitted helminth infections, much attention is not given to *Strongyloidiasis* by the policymakers although the global burden is probably much higher than previously estimated. We encourage researchers to work on standardizing diagnostic protocols of *strongyloidiasis* and also policymakers to include s*trongyloidiasis* in the soil-transmitted helminth package.

### 4.1. Limitation of This Review

The use of only PubMed and Google Scholar databases as a source of articles was the limitation of this review.

## 5. Conclusions

This review shows that s*trongyloidiasis* prevalence is overlooked and its prevalence is low in Africa due to the use of low-sensitivity diagnostic methods and lack of correct diagnostic approach. A combination of microscopic and PCR method gives good detection rate of s*trongyloidiasis*. Therefore, there is a need for using a combination of microscopic and molecular-based diagnostic methods to determine the true prevalence in Africa. Further research is also needed to break the transmission cycle and reduce the impacts of s*trongyloidiasis* in the African population.

## Figures and Tables

**Figure 1:** Overview of search methods of article inclusion and exclusion criteria.

**Figure 2:** Forest plot of strongyloidiasis in African countries using random effects model.

**Figure 3:** Forest plot of strongyloidiasis prevalence by diagnostic methods using random effects model.

**Figure 4:** Forest plot of strongyloidiasis prevalence by study settings using random effects model.

**Figure 5:** Forest plot of strongyloidiasis prevalence among patients using random effects model.

**Figure 6:** Funnel plot displaying strongyloidiasis prevalence data for all included publications.

**Table 1:** The main characteristics of the included articles.

Authors' information and reference	Diagnostic methods	Study settings	*S. stercoralis* Pos (*n*, %)	Sample size
Dacal et al., 2018, Angola [19]	PCR	School	75 (21.4)	351
Bocanegra et al., 2015, Angola [20]	FECT	School	1 (0.07)	1425
de Alegrıa et al., 2017, Angola [21]	BCT, FECT	School	28 (12.2)	230
Karou et al., 2011, Burkina Faso [22]	DSM	H/institution	6 (0.05)	11,728
Bopda et al., 2016, Cameroon [23]	KK	H/institution	7 (2.1)	334
Nsagha et al., 2016, Cameroon [11]	FECT	H/institution	2 (0.7)	300
Kuete et al., 2015, Cameroon [24]	FECT	H/institution	4 (0.9)	428
Becker et al., 2015, Côte d'Ivoire [25]	BCT, culture, PCR	Community	56 (21.9)	256
Glinz et al., 2010, Côte d'Ivoire [26]	BCT, culture	School	68 (27.1)	251
Rayan et al., 2011, Egypt [27]	BCT, FECT, culture, PCR	H/institution	18 (15.7)	115
Roka et al., 2013, Equatorial Guinea [28]	FECT	H/institution	28 (10.3)	273
Roka et al., 2012, Equatorial Guinea [29]	FECT	H/institution	23 (8.8)	260
Amor et al., 2016, Ethiopia [6]	BCT, FECT, PCR	School	82 (20.7)	396
Abdia et al., 2017, Ethiopia [30]	FECT	School	3 (0.7)	408
Ramos et al., 2014, Ethiopia [31]	DSM	H/institution	92 (0.3)	32191
Zeynudin et al., 2013, Ethiopia [32]	FECT	H/institution	6 (6.6)	91
Assefa et al., 2009, Ethiopia [33]	FECT	H/institution	28 (7.4)	378
Wegayehu et al., 2013, Ethiopia [34]	FECT	Community	51 (5.9)	858
Huruy et al., 2011, Ethiopia [35]	DSM	H/institution	12 (3.1)	384
Gedle et al., 2015, Ethiopia [36]	FECT	H/institution	5 (1.6)	305
Abera et al., 2013, Ethiopia [37]	FECT	School	27 (3.4)	788
Derso et al., 2016, Ethiopia [38]	DSM	H/institution	6 (1.6)	384
Fekadu et al., 2013, Ethiopia [39]	FECT	H/institution	36 (10.5)	343
Abate et al., 2013, Ethiopia [40]	FECT	H/institution	8 (2.0)	410
Alemu et al., 2017, Ethiopia [41]	FECT	H/institution	4 (1.8)	220
Teklemariam et al., 2013, Ethiopia [42]	FECT	H/institution	15 (4.0)	371
Legesse et al., 2010, Ethiopia [43]	FECT	School	1 (0.3)	381
Hailu et al., 2015, Ethiopia [44]	FECT	H/institution	5 (0.05)	100
Nyantekyi et al., 2010, Ethiopia [45]	FECT	Community	38 (13.2)	288
Chala, 2013, Ethiopia [46]	DSM	H/institution	73 (1.2)	6342
M'bondoukwé et al., 2018, Gabon [47]	DSM	Community	10 (3.7)	270
Janssen et al., 2015, Gabon [48]	Culture	H/institution	10 (4.0)	252
M'bondoukwé et al., 2016, Gabon [49]	DSM	H/institution	1 (1.0)	101
Adu-Gyasi et al., 2018, Ghana [50]	FECT	Community	14 (0.9)	1569
Nkrumah et al., 2011, Ghana [51]	DSM	Hospital	6 (0.6)	1080
Forson et al., 2017, Ghana [52]	FECT	School	1 (0.3)	300
Yatich et al., 2009, Ghana [53]	BCT	H/institution	29 (3.9)	746
Sam et al., 2018, Ghana [54]	FECT	School	20 (5.1)	394
Cunningham et al., 2018, Ghana [55]	PCR	Community	5 (1.1)	448
Kagira et al., 2011, Kenya [56]	DSM	H/institution	3 (9.7)	31
Walson et al., 2010, Kenya [57]	FECT	Community	20 (1.3)	1541
Arndt et al., 2013, Kenya [58]	FECT	Community	5 (3.3)	153
Meurs et al., 2017, Mozambique [59]	FECT, BCT, PCR	Community	147 (48.5)	303
Cerveja et al., 2017, Mozambique [60]	DSM	H/institution	5 (1.3)	371
Chukwuma et al., 2009, Nigeria [61]	FECT	School	13 (5.9)	220
Uhuo et al., 2011, Nigeria [62]	FECT	School	4 (0.5)	800
Wosu and Onyeabor, 2014, Nigeria [63]	FECT	School	11 (3.6)	304
Simon-oke et al., 2014, Nigeria [64]	DSM	School	23 (12.8)	180
Adekolujo et al., 2015, Nigeria [65]	FECT	H/institution	4 (0.6)	717
Olusegun et al., 2011, Nigeria [66]	DSM	School	2 (0.7)	304
Abaver et al., 2011, Nigeria [67]	FECT	H/institution	3 (2.5)	119
Ivoke et al., 2017, Nigeria [68]	FECT	H/institution	8 (1.0)	797
Ojurongbe et al., 2018, Nigeria [69]	FECT	H/institution	2 (1.0)	200
Emeka, 2013, Nigeria [70]	FECT	School	28 (11.0)	255
Esiet and Edet, 2017, Nigeria [71]	FECT	School	46 (4.4)	1055
Manir et al., 2017, Nigeria [72]	FECT	School	10 (4.0)	252
Onyido et al., 2016, Nigeria [73]	FECT	School	1 (0.8)	120
Abah and Arene, 2015, Nigeria [74]	FECT	School	273 (7.1)	3826
Damen et al., 2010, Nigeria [75]	FECT	School	34 (6.8)	500
Akinbo et al., 2010, Nigeria [76]	FECT	H/institution	23 (1.2)	2000
Ojurongbe et al., 2014, Nigeria [77]	FECT	School	6 (3.7)	162
Amoo et al., 2018, Nigeria [78]	FECT	H/institution	10 (4.3)	231
Alli et al., 2011, Nigeria [79]	FECT	H/institution	4 (1.1)	350
Eke et al., 2015, Nigeria [80]	FECT	School	63 (13.1)	480
Auta et al., 2013, Nigeria [81]	FECT	School	12 (4.2)	283
Aniwada et al., 2016, Nigeria [82]	FECT	School	10 (1.2)	859
Umar and Bassey et al., 2010, Nigeria [83]	Culture	School	104 (37.1)	280
Tuyizere et al., 2018, Rwanda [84]	Culture	Community	94 (17.4)	539
Ferreira et al., 2015, Sao Tome and Principe [85]	FECT	Community	11 (2.5)	444
Sow et al., 2017, Senegal [86]	PCR	H/institution	6 (6.1)	98
Babiker et al., 2009, Sudan [87]	FECT	H/institution	2 (0.1)	1500
Mohamed et al., 2018, Sudan [88]	DSM	H/institution	1 (0.2)	600
Knopp et al., 2014, Tanzania [89]	BCT, PCR	Community	83 (7.4)	1128
Salim et al., 2014, Tanzania [90]	BCT	Community	71 (6.9)	1033
Sikalengo et al., 2018, Tanzania [91]	BCT	H/institution	89 (13.3)	668
Mhimbira et al., 2017, Tanzania [92]	BCT, FECT	Community	161 (16.6)	972
Barda et al., 2017, Tanzania [93]	BCT, culture	School	36 (7.1)	509
Oboth et al., 2019, Uganda [94]	KK	Refuge	1 (0.2)	476
Stothard et al., 2008, Uganda [95]	BCT	Community	4 (1.3)	301
Hillier et al., 2008, Uganda [96]	BCT	Community	256 (12.4)	2059
Kelly et al., 2009, Zambia [97]	DSM	Community	14 (0.5)	2981
Knopp et al., 2008, Zanzibar [98]	BCT, culture	Community	7 (2.2)	319
*Total*			**2614 (2.7)**	**96,069**

^∗^BCT = Baermann concentration technique; DSM = direct saline microscopy; FECT = formol ether concentration technique; H/institution = health institution; KK = Kato-Katz; PCR = polymerase chain reaction.

## Data Availability

The data can be requested from Bahir Dar University (https://bdu.edu.et/node/74).
